The article "Construction of Sports and Health Data Resources and Transformation of Teachers' Orientation Based on Web Database" was retracted in 2023. Reasons: suspected computer-generated content; unreliable results or conclusions; concerns about the data; concerns about the results or conclusions.

# Construction of Sports and Health Data Resources and Transformation of Teachers' Orientation Based on Web Database

**DOI:** 10.1155/2022/4372406

**Published:** 2022-02-07

**Authors:** Jiawen Yang, Min Chen

**Affiliations:** ^1^College of Physical Education and Health Science, Chongqing Normal University, Chongqing 401331, China; ^2^School of Physical Education, Yulin Normal University, Yulin, Guangxi 537000, China

## Abstract

In the intelligent era, emerging information technology helps to transform the information society into an intelligent society and the educational system into a new educational ecology. Teachers must change their roles to be competent for future education and teaching as a result of social transformation, technology application, and education development. Simultaneously, figuring out how to sort sports health data and analyze students' physical health information with a low error rate is an urgent problem that needs to be solved. Data management skills are an unavoidable requirement of the current state of school physical education. Sports health information management will become easier as computer technology advances and the country places a greater emphasis on computer networks. This paper proposes a Web database-based sports health data management system. This paper can help schools understand the relationship between important factors and indicators that affect students' health in order to guide them in making timely changes to their physical education programs. Provide a reasonable sports health plan based on scientific analysis and evaluation to achieve the goal of improving students' physical quality and reducing workload.

## 1. Introduction

With the gradual improvement of living standards, various factors such as unhealthy lifestyles directly threaten people's health, and the reason is that people's awareness and concept of personal health management are weak [1]. In daily life, there are many benefits of sports. It can enhance people's ability to resist diseases, and enhance various physical functions and potentials [2]. Moderate exercise can make you happy physically and mentally, relieve the pressure brought about by work and troubles, prevent various mental problems caused by psychological disorders, and add a lot of happiness to your life. Therefore, exercise is an important part of health management, which can bring personal health [3]. Based on this, it is imperative to strengthen modern people's personal health management, develop good habits of sports health, and implement scientific and reasonable sports health management. Sports health management is the management process of people's self-health risk factors, and it has been paid more and more attention in the world [4]. With the continuous expansion of the scale of college students in China, the number of students increases rapidly, so the anthropometric data related to students also increases significantly, including student attendance information and physical health test data [5]. In the manual management of a large amount of information, mistakes often occur, which easily affect the enthusiasm of students to participate in sports and fail to achieve the purpose of urging students to exercise [6]. At the same time, it also brings many adverse effects to some schools to carry out sports activities. Therefore, how to conveniently and efficiently sort out sports health data and analyze students' physical health information with low error rate is an urgent problem to be solved. Doing a good job in data management is the inevitable requirement of the current development of school physical education.

The article "Construction of Sports and Health Data Resources and Transformation of Teachers' Orientation Based on Web Database" was retracted in 2023. Reasons: suspected computer-generated content; unreliable results or conclusions; concerns about the data; concerns about the results or conclusions.

With the constant awakening of people's health awareness, the sports health system has generated more and more information, including students' sports information and students' physical health test data. Then, doing a good job in data management is the inevitable requirement of current development. Physical education and health course takes physical exercises as the main means and aims at improving students' health [7]. It adheres to the guiding ideology of “health first,” takes students' development as the center, and always puts students' active development in a prominent position. Through rich and colorful sports activities, students' interest in sports is stimulated and their awareness of lifelong sports is cultivated [8]. The curriculum of physical education and health has changed from the direction of the organic combination of physical education and education, and the organic connection between physical education and health. Whether this idea and conception can be really implemented and they achieve the expected results depends on the concrete implementer-physical education teachers, the role played by physical education teachers in school education, and their understanding and understanding of their own roles [9]. For a long time, society has held the belief that physical education teachers should play a role. PE teachers have gradually formed their own role orientation, restricting their thoughts and behaviors with this role, influenced by societal expectations and their role consciousness—the role of their knowledge, attitude, and behavior tendency [10]. Teachers in the new era should consider the benefits and drawbacks of the new era and complete their own role positioning. As a result, research into the role orientation of physical education teachers in school physical education to promote sports and health is critical. Many schools are currently dealing with the issue of sloppy multi-campus sports health management [11]. To make sports health data management efficient and intelligent, it is necessary to research and develop a comprehensive sports health management system combined with modern network technology in order to better carry out school physical education. This paper summarizes the working principle of a World Wide Web (Web) database, proposes a sports and health data resource system based on a Web database, and describes the implementation process based on the development of management information systems.

The article "Construction of Sports and Health Data Resources and Transformation of Teachers' Orientation Based on Web Database" was retracted in 2023. Reasons: suspected computer-generated content; unreliable results or conclusions; concerns about the data; concerns about the results or conclusions.

A complete health plan should include three aspects: exercise, diet, and health guidelines. Sports health management is an important part of health management, and physical testing is an important link of sports health testing [12]. Exercise prescription is the process of reasonably guiding and formulating exercise plan according to various exercise test results. Give full play to the advantages of computer network technology, introduce it into modern sports health management, actively build an interactive platform for sports health management based on Web database technology, meet the sports health needs of the public, provide personalized physical fitness assessment, provide special sports health programs, and improve personal sports health level, It is an important content of personal health management [13]. This paper constructs student sports and health data resource database and video database based on Web database. The students' sports, health data, physique monitoring, and methods and means of improving students' physique are systematized and shared with information, so as to improve the tedious work of students' physique monitoring. Strive to improve the diversification and scientification of methods and means of students' physique, reduce the error probability of students' physique monitoring, improve students' physique work, and reduce the workload.

## 2. Related Work

According to the literature [14], users can log in to different database servers; select different authentication methods and log in users; and perform database, data table, and data view operations by designing and implementing a user database resource management system based on the Web. According to the literature [15], exercise prescription is the most common method of exercise health management. It is a healthy exercise program that is tailored to each person's specific needs. This method is quantitative, and the exercise mode is chosen with medical and health knowledge in mind. Literature [16] developed a Web database-based sports health management platform, created and adjusted intelligent sports prescriptions, and used information technology to assist people in improving their physical conditions. According to the literature [17], Internet users retrieve information using a unified web interface, which is less expensive than client software for document management systems and groupware. The combination of this integrated information network system database and web server has spawned a new area of Internet development for the next generation. According to literature [18], in order to be competent for future education and teaching, teachers must change their roles and reposition their work content from the dimensions of education and teaching, learning service, technology application, and subject attribute. According to literature [19], the core content of the construction of a sports health management platform is to create a networked and efficient personal sports health evaluation system as well as a personalized exclusive sports health scheme system. Literature [20] proposes that, thanks to the rapid development of Browser/Server structure (B/S), more and more software engineers began to focus on the design and development of Web applications. The load of client computers was greatly reduced, and the cost and workload of system maintenance and upgrading were reduced. Literature [21] in sports health management gives full play to the advantages of ASP technology and B/S structure technology, and establishes a scientific, practical, simple, and extensible sports health management platform based on Web database technology. Literature [22] proposed that when creating web pages and developing web database pages, first we should establish some static hypertext markup language (HTML) pages that support the whole web file system. We can also use InterDev to add files to them. Literature [23] considered that the application system based on Web development is a one-step development, which can enable different operators to access and operate the common database in different access ways from different places, and can effectively protect the server data platform. Literature [24] starts with the role orientation of teachers in the intelligent era, puts in perspective the demands of teachers' literacy in the intelligent era, and then constructs the framework of teachers' intelligent education literacy, so as to provide reference for teachers' training and normal students' training. In literature [25], the Web-based user database resource management system is designed and implemented akin to the three-layer MVC architecture. The responsibilities and functions of each level are very clear, which greatly improves the scalability and maintainability. The developed system components have strong reusability and strong universality, which provides convenience for later transplantation to other management systems. Literature [24] discusses the transformation of teachers' role in the era of intelligence from four aspects. Based on the perspective of four dimensions, combined with the development and evolution of educational objectives, educational environment, and educational activities in the intelligent era, this paper combs the specific direction of teachers' role transformation in the future. Literature [26] mentioned that the Web is a global, interactive, dynamic, multi-platform and distributed graphic information system based on the Internet. It is an important means of retrieving information on the Internet. This paper designs and implements the student sports and health data resource management system. This system realizes the open and ecological linkage output of exercise and nutrition prescription, and makes the exercise video, which improves individual compliance. Combined with the analysis of sports data, the transfer progress degree of group exercise is obtained. Compared with the results of the traditional average evaluation method, it is found that the system can eliminate the differences in physical basis of individuals within the group and achieve a more fair and reasonable health evaluation of sports groups.

The article "Construction of Sports and Health Data Resources and Transformation of Teachers' Orientation Based on Web Database" was retracted in 2023. Reasons: suspected computer-generated content; unreliable results or conclusions; concerns about the data; concerns about the results or conclusions.

## 3. Methodology

### 3.1. Design and Implementation of Web Database

With the rapid growth of the Internet, the combination of database and network technology is becoming more and more common, and the development mode of network applications has shifted from C/S to B/S architecture. The question of how to create a reliable and efficient Web-based user database resource management system has risen to prominence in the field of information technology research [27]. At the same time, remote database resource management is realized, making database resource management more convenient for users.

At present, the integration schemes and technologies of Web and database are very complicated, which can be roughly divided into three categories. One is the technology developed by database manufacturers. Second, the technology developed by intermediate manufacturers. Third, the technology provided by Web server developers. The realization of various methods can be summarized as follows: the browser is used as the container for downloading the homepage from the Web server, the user fills in the query information in the form and gives it to the server, the server interfaces with the external database in different ways, runs the operations such as query and update, returns the operation results to the server, and formats them into HTML pages and then sends them to the client browser.

The article "Construction of Sports and Health Data Resources and Transformation of Teachers' Orientation Based on Web Database" was retracted in 2023. Reasons: suspected computer-generated content; unreliable results or conclusions; concerns about the data; concerns about the results or conclusions.

Web database is mainly composed of four parts, that is, the design of HTML, Web editing language, common gateway interface (CGI), and database backend. The application of Web database consists of three parts: Web server, network database, and users [28]. Generally, the Web server and CGI external application exist on one host at the same time, while the database server and the Web server can be set up on one host at the same time or on two different hosts, respectively. From a technical point of view, there are four ways to realize the connection between Web and database. ① Use common gateway interface public gateway interface. ② Create a connection from the public gateway interface to the open database connection interface. ③ Use the Web server extension software to access the remote database. ④ Use a Web server with ODBC interface.

The working process of Web database is actually a CGI application process. The whole working principle can be roughly divided into five parts. ① From users to Web servers. ② From Web server to CGI external program. ③ CGI external program and database server. ④ From CGI external program to Web server. ⑤ From Web server to user. The Web server uses HTML language to return data to users in a specific form, and then completes an access operation to the Web server. The process is shown in Figure 1.

This sports health data management system uses a mature B/S architecture, which it effectively combines with the development of a Web database to create a three-tier B/S architecture. The sports network management system is developed using ASP technology, which combines the sports management and network platform. The data warehouse technology is introduced, and an innovative analysis module is added to analyze sports management results, provide timely feedback, and seek out the best management mode. In data management query, new methods of multi-keyword query and fuzzy query are introduced. In general, it meets the requirements for a sports network management system's development and is technically feasible. Web applications have obvious advantages over traditional desktop applications, including ease of development, installation, and post-maintenance, as well as a large user base [29]. Generally speaking, in a Web application, when a user submits a form, the server will accept the whole form and forward it to the script that processes the form, and then send a brand-new page back to the user after execution. The overall functional module structure diagram of the Web system in this paper is shown in Figure 2.

The article "Construction of Sports and Health Data Resources and Transformation of Teachers' Orientation Based on Web Database" was retracted in 2023. Reasons: suspected computer-generated content; unreliable results or conclusions; concerns about the data; concerns about the results or conclusions.

The problem to be solved in the realization of Web database is to configure the Web information server on IIS under the NTServer. At the back end of the database, create the network database with the SQLServer, and connect the Web with the network database with development tools, so as to realize the Web database. The core of the problem is how to realize the connection between Web and database. The server data (stored in the Web form) is returned to JavaScript code, which can quickly update the form data, and users can hardly feel any delay, and get new data without refreshing or submitting. The power of HttpRequest lies in this: it can interact with the server on its own according to needs, and users can even do everything without knowing the background at all. This is a dynamic, fast response, and highly interactive experience similar to desktop applications, and it also integrates the powerful power of the Internet.

### 3.2. Teacher Orientation Change

Emerging information technologies, such as artificial intelligence and virtual reality, are accelerating the transition to an intelligent society, resulting in shifts in talent demand. They are also remaking the learning environment and causing changes in the teaching process at the three levels of perception, knowledge, and cognition, paving the way for the development of human-computer collaborative teaching. Teachers will face new challenges as future education is reconstructed and reformatted. Teachers' roles must change and develop in the age of intelligence, taking into account aspects of education and teaching, learning and service, technology application, and subject attributes. Teachers must have technology cognition literacy, innovative teaching, human-computer cooperation, resource integration, data application, ethical security, and other skills. Under the influence of traditional educational ideas, physical education teachers' role orientation has been in conflict with the role that physical education teachers should play under the guiding ideology of the Physical Education and Health Curriculum Standard, which appears out of place and leads to the phenomenon of dislocation of physical education teachers' roles in long-term practice of school physical education.

With the transformation of social productivity and form caused by the application of intelligent technology, the training of talents in the education system needs to meet the needs of social talents, and pay attention to the cultivation of higher-order thinking and accomplishment of learners to cope with future social life and professional challenges. At the same time, the in-depth application of intelligent technology in the education system will also lead to the changes of teaching environment, teaching activities, teaching modes, learning methods, management methods, etc., and promote the changes of educational subject view, educational communication view, and knowledge view, and help the systematic reform and reshaping of educational ecology. These changes will lead to the reconstruction of teachers' future professional division and orientation, and promote the transformation of teachers' roles. Under the new curriculum standard, PE teachers become promoters of PE teaching and researchers of education and teaching activities accordingly.

The article "Construction of Sports and Health Data Resources and Transformation of Teachers' Orientation Based on Web Database" was retracted in 2023. Reasons: suspected computer-generated content; unreliable results or conclusions; concerns about the data; concerns about the results or conclusions.

Education in the era of intelligence requires teachers to have intelligent education literacy covering technology, education, and society; fully understand the nature, logic, enablement, and possibility of technology; innovatively design and implement human-computer collaborative education and teaching activities; and fully understand and respond to social risks and professional challenges brought about by technology application. As a promoter of sports health, physical education teachers' roles and behaviors are as follows: helping students decide appropriate learning goals, and confirming and coordinating the best way to achieve these goals; guiding students to form good study habits, master learning strategies, and cultivate the ability to exercise independently; creating rich teaching situations, stimulate students' learning motivation, cultivate their interest in learning and fully mobilize their learning enthusiasm; and providing various convenient services for students' study.

The change of teacher's role from the perspective of education mainly focuses on the change of teacher's teaching purpose, content, and method. At the level of teaching purpose, intelligent technology promotes the development of social productive forces, the transformation of industrial structure, and the reorganization of human-machine division of labor, which in turn creates new demands for the cultivation of educational talents and forces teachers to change their teaching. In school physical education, the teaching concept of competitive sports has been favored for a long time. At the technical level, the goal of school physical education is more defined, and the physical education teacher completely transforms into a coach engaged in sports technical training. Students have high expectations for establishing and maintaining a new teacher-student relationship with physical education teachers, according to the research. Teachers should be skilled at providing students with a sense of psychological safety and spiritual encouragement in a variety of ways, in order to stimulate their thinking and increase their exploration enthusiasm; actively create a learning environment for students; when exercises fail or movements are not standardized, teachers should understand and encourage them, in order to create a safe learning environment and promote their continuous exploration and thinking.

The article "Construction of Sports and Health Data Resources and Transformation of Teachers' Orientation Based on Web Database" was retracted in 2023. Reasons: suspected computer-generated content; unreliable results or conclusions; concerns about the data; concerns about the results or conclusions.

In the aspect of knowledge transmission, teachers will turn from instigator to guide, paying attention to inspiring and assisting learners' independent knowledge construction and cognitive development. In the aspect of educating people, education and teaching in the intelligent age pay more attention to the cultivation of learners' ability, wisdom enlightenment, and individual potential stimulation, and the cultivation of learners' higher-order rational thinking ability, interactive thinking, and lifelong learning ability. In terms of teaching content, teachers are no longer teaching based on specific textbooks and specific contents. They need to design and develop thematic and modular courses according to students' learning situation and needs, combined with various resources, and become teaching designers and planners. At the level of teaching methods, teachers need to pay more attention to the support and precise guidance of learners' learning process, and give full play to students' learning initiative. With the implementation of the new curriculum in the context of quality education, the problems in the educational situation have greatly increased and become very complicated. Therefore, the requirement of “teachers are researchers” is particularly important in the context of the new curriculum. Teachers must gradually develop the consciousness and ability of self-reflection, scientific design of education and teaching behaviors, and engaging in educational action research, which is not only the need of the development of quality education, the need of promoting students' development, but also the need of teachers' self-development.

Physical education teachers should be fully aware that they are not only a coach engaged in sports technical training but also a real educator who can cultivate students' sound personality and healthy psychology, and promote their all-round development. Physical education teachers should not only pay attention to the teaching of basic knowledge and sports skills of sports and health, the exercise of sports skills and skills, and the development of students' physical quality and physical function but also impart scientific outlook on life and values to students, and guide students to form a good ideological style and attitude towards life.

The article "Construction of Sports and Health Data Resources and Transformation of Teachers' Orientation Based on Web Database" was retracted in 2023. Reasons: suspected computer-generated content; unreliable results or conclusions; concerns about the data; concerns about the results or conclusions.

### 3.3. Construction of Sports and Health Data Resource System

Sports health management is a new health concept and health management method in recent years. It is mainly to scientifically and reasonably formulate some sports prescriptions according to users' sports data and natural conditions, and the ultimate goal is to improve users' health and physical fitness. Sports health management system has developed to a great extent in foreign countries, and it is increasingly accepted by the masses in China. At present, companies and institutions related to health management are constantly being established in China, but the construction of health management system in Chinese schools is still not to the desire level. According to the survey, at present, school students' awareness of physical health management is generally lacking.

The sports health management system described in this paper has several obvious advantages over traditional management methods, including the following: Modern Web technology can enable cross-platform message publishing and information browsing, as well as dynamic interactive management, thanks to advancements in computer network technology. Sports health management can be accomplished using network technology, computer technology, and database technology. The sports health data management platform is built and implemented using Web database technology, with ASP, HTML, and other web page programming languages and database technology serving as the primary technical support. Its network environment is primarily supported by the Internet, and unified management of individual sports health is realized using FTP tools, allowing users to access remote and personalized sports health services. Users can not only make requests but also receive Web information via the Web browser.

In the scheduling of fitness benefit index heterogeneous data information resources, s_*j*_^(k)^ and y_*j*_^(k)^ are used to represent the linear input and reversible invariance output of the system, and the feature vector is expressed as:

(1) $$\begin{array}{c} x^{\left(k\right)}={\left[x_{1}^{\left(k\right)},x_{2}^{\left(k\right)},\ldots ,x_{N_{k-1}}^{\left(k\right)}\right]}^{T}, \end{array}$$

(2) $$\begin{array}{c} s^{\left(k\right)}={\left[s_{1}^{\left(k\right)},s_{2}^{\left(k\right)},\ldots ,s_{N_{k}}^{\left(k\right)}\right]}^{T}, \end{array}$$

(3) $$\begin{array}{c} y^{\left(k\right)}={\left[y_{1}^{\left(k\right)},y_{2}^{\left(k\right)},\ldots ,y_{N_{k}}^{\left(k\right)}\right]}^{T}. \end{array}$$

The time-frequency characteristics of cardiopulmonary function data under comprehensive fitness are to be studied, so as to use the characteristics as the medium to reflect the original characteristics of the cardiopulmonary function data. Suppose the value range of the range data is N discrete points A={a_1_,…,a_N_}, then the time average value of the national fitness benefit index is calculated as follows:

(4) $$\begin{array}{c} t_{m}=\frac{1}{E_{x}}\int_{-\infty }^{+\infty }t{\left|x\left(t\right)\right|}^{2}\mathrm{dt}. \end{array}$$

Frequency mean:

(5) $$\begin{array}{c} \upsilon_{m}=\frac{1}{E_{x}}\int_{-\infty }^{+\infty }\upsilon {\left|X\left(\upsilon \right)\right|}^{2}d\upsilon . \end{array}$$

The fitness benefit index system based on linear model or equivalent approximation is obtained.

The article "Construction of Sports and Health Data Resources and Transformation of Teachers' Orientation Based on Web Database" was retracted in 2023. Reasons: suspected computer-generated content; unreliable results or conclusions; concerns about the data; concerns about the results or conclusions.

The key technology of the sports health management platform is database technology. The platform's purpose is to extract, analyze, and process a large amount of data before providing feedback to customers. The database can perform data sorting and simple analysis on its own, and as a development tool, it can perform secondary development and data maintenance more quickly. To achieve data management, a database must design a large number of tables, for example, a user information table, a statistical information table, and so on. User name, gender, sports content, sports time, sports frequency, and sports intensity are all needed in the user information table. The five elements of exercise health management are represented as data items in the exercise prescription table, and each data table is linked by user name to enable basic keyword queries and facilitate feedback on reasonable exercise prescriptions. The relationship table between sports and diseases, in particular, must be designed in a one-to-many or one-to-one data storage mode, and these critical medical care data must be stored in a server that is easy to query and call.

Combine the weekly average energy consumption sequence of all exercise individuals for two consecutive weeks into one observation sequence, and first find the minimum value (e_min_) and maximum value (e_max_) of the sequence. Based on this, *m* state intervals are divided, and the span of each interval is Δe = (e_max_  −  e_min_)/m, then the state interval of the energy consumption sequence is as follows:

(6) $$\begin{array}{c} \left[e_{\min},e_{\min}+\Delta e\right],\ldots ,\left[e_{\min}+\left(m-1\right)\cdot \Delta e,e_{\max}\right]. \end{array}$$

According to the transition probability matrix, the transition progress of the current Markov chain can be calculated:

(7) $$\begin{array}{c} K=\sum_{i=1}^{m}\sum_{j=1}^{m}{\left(j-1\right)}^{3}\cdot p_{ij},i,j\in \left[1,m\right]. \end{array}$$

After calculating the transfer progress degree of sports energy consumption of each group, respectively, it is used as the health evaluation model of sports groups to compare the exercise effects of sports groups.

The article "Construction of Sports and Health Data Resources and Transformation of Teachers' Orientation Based on Web Database" was retracted in 2023. Reasons: suspected computer-generated content; unreliable results or conclusions; concerns about the data; concerns about the results or conclusions.

The programming language for the sports health management platform is ASP, which stands for dynamic server page. AetiveX components work with ASP instructions to build Web server applications through an organic combination of HTML pages and ASP. Simultaneously, it can ensure that the application program is effective, interactive, and simple to use. The use of an ASP application in conjunction with HTML code and a scripting language can ensure that the ASP program runs safely and that the ASP source code is not transmitted to the client, which has strong applicability characteristics.

Build a nonlinear dynamic system that can fit many influencing factors, and realize the fitting of a benefit index parameter system. The fitting model is described as follows:

(8) $$\begin{array}{c} {\text{R}}_{\beta }\text{X}=\text{U}\left\{\text{E}\in \text{U/R}|\text{c}\left(\text{E,X}\right)\leq \beta \right\}, \end{array}$$

(9) $$\begin{array}{c} {\text{R}}_{\beta }\text{X}=\text{U}\left\{\text{E}\in \text{U/R}|\text{c}\left(\text{E,X}\right)\leq 1-\beta \right\}, \end{array}$$

(10) $$\begin{array}{c} {\text{bnr}}_{\beta }\left(\text{X}\right){=\text{R}}_{\beta }{\text{X}-\text{R}}_{\beta }{\text{X}}_{1}. \end{array}$$

It is necessary to include the universal influence factor group, and select the number of principal components according to the contribution degree of cumulative variance. Only when the cumulative contribution rate reaches a certain amount, the corresponding *m* principal components can be selected as the principal components. The above fractal design provides accurate resource data basis for realizing a heterogeneous data mining model of sports health benefit index.

The development and design of a sports health management platform based on Web database technology adheres to the personal health management principle of “prevention first, sports intervention.” We can work out the exercise mode suitable for individuals using the personal sports health plan module and the health information table, which we can combine with the specific characteristics of different groups of people. The sports data management platform's main functions include not only adjusting physical diseases and recovering quickly but also preventing diseases. Sports health management is a networked health management platform that selects sports methods and contents based on people's characteristics, according to relevant scientific data.

## 4. Results Analysis and Discussion

Sports health management is a systematic project. Today, with the development of information network technology, we should give full play to its advantages and introduce it into the field of student health management. Actively establish the platform of sports health management system, strengthen personal sports health management, and improve students' sports health quality, so as to change health management from passive to active, and comprehensively improve students' health level. Abundant sports data can be generated in the process of exercise. By analyzing these sports data, we can find out the rules of people in the process of exercise. If the sports data are combined with the athletes' own physical fitness indexes for analysis, the physical health in the process of exercise can be evaluated.

The article "Construction of Sports and Health Data Resources and Transformation of Teachers' Orientation Based on Web Database" was retracted in 2023. Reasons: suspected computer-generated content; unreliable results or conclusions; concerns about the data; concerns about the results or conclusions.

According to the research, there is a certain gap in health status between students who participate in health management and those who do not. From the results of the experimental intervention group and the control group in Figure 3, it can be seen that the health status of the students who participated in health management has improved to some extent compared with those who did not participate in health management.

The ASP, B/S architecture, and Web database technology are used to create the sports health management platform described in this paper. Customers' sports health is managed and exercise prescriptions are given using a networked platform. Both unhealthy and healthy students are to be assisted in improving their physical condition. The platform's development language is ASP, which is a dynamic web page technology, and some common functions can be accomplished with HTML code. ActiveX controls can also be used by ASP to access users' sports health data. ASP has good interactive performance, can be used with a variety of software, and includes some built-in objects that can easily enhance the server's script function, allowing data uploaded by users to be further processed and stored in real time. The weight can be adjusted adaptively in this algorithm to achieve adaptive convergence, which improves the controllability and universality of the algorithm retrieval and data mining performance. The convergence curve of this algorithm is shown in Figure 4.

By analyzing the above experimental results, we can see that through heterogeneous data mining of the fitness benefit index, we get the promotion relationship model of sports health training for students' health benefit index, and master the improvement degree of fitness exercise for different groups' physical functions. Compared with traditional methods, the accuracy of this method is improved and the robustness is better.

The article "Construction of Sports and Health Data Resources and Transformation of Teachers' Orientation Based on Web Database" was retracted in 2023. Reasons: suspected computer-generated content; unreliable results or conclusions; concerns about the data; concerns about the results or conclusions.

After the user requests from the network enter the system, they are placed in a request task queue, waiting for the system to assign threads to execute. This request task queue is blocked, which can reduce the pressure on the server when the user requests too much. Access to shared resources with the system is protected by synchronization. In the multithreading concurrency model, the execution of each user request has gone through a complete set of processes: accepting the request, assigning the thread to perform the task, and returning the processing result. The processing logic of this model is clear, and a complete request processing logic can be put together, which simplifies the development. Moreover, due to the introduction of threads, the processing of requests has good isolation. In addition, the synchronization mechanism is used to access shared resources, which ensures the consistency of the system.  Figure 5 shows that the performance of multithreaded concurrent server is affected by the change of the thread number.

System programming allows for logical control of the questionnaire and data, the avoidance of logical errors and abnormal values in the questionnaire data, and the assurance of data quality. However, in the design and application of this platform, it is worth noting that, in the case of a large amount of user data, databases such as Oracle or SQLServer are preferable to access databases in terms of practical performance. Because exercise intensity has a direct impact on human health, we can assess exercise health by examining exercise intensity changes. The expression of exercise intensity varies depending on the type of exercise. In this paper, we use a unified evaluation index to measure exercise intensity during exercise using a variety of sports data, laying the groundwork for future research into sports health evaluation models.

When all connections are established and sent, the timer starts. At this time, all connections start to send requests at the same time, and the timer stops after the last connection request receives a response, so as to calculate the number of connection requests that the server can handle per second under different concurrent connections. The test results are shown in Figure 6.

The student health management system has played a certain and positive role in improving students' health. However, due to the limited management time and the influence of many factors, the multi-directional and three-dimensional management system failed to show its full effectiveness, and the implementation of intervention measures failed to maximize, comprehensively and continuously. Therefore, there is no significant difference in individual items. This suggests that we need to continue to carry out sustainable health management for students. The comparison of the limit energy consumption rate and the energy consumption rate of athletes in each time period is shown in Figure 7.

The article "Construction of Sports and Health Data Resources and Transformation of Teachers' Orientation Based on Web Database" was retracted in 2023. Reasons: suspected computer-generated content; unreliable results or conclusions; concerns about the data; concerns about the results or conclusions.

From Figure 7, it can be found that since the 1100s, the athlete's energy consumption rate began to be lower than the limit energy consumption rate, and it continued to decrease with time. This indicates that his or her physical strength is beginning to decline. At this time, he or she should be advised to gradually reduce the intensity of exercise or stop exercising to have a rest, so as to ensure the benefit of exercise and minimize the occurrence of danger.

As for the health evaluation of sports groups, because of the differences in individual physical foundations within sports groups, only the average value of group sports result data is used to reflect the improvement degree of group exercise effect, without considering the individual differences within groups, which cannot reflect the actual exercise effect of groups. Therefore, the sports group health evaluation model is based on Markov model, which calculates the data changes of two sports exercises of the group. This paper proposes to use the transfer progress degree to evaluate the improvement degree of sports exercise effect. Through the experiment, the errors produced by the sports individual health evaluation model in evaluating each sports individual are calculated, and the errors are plotted. The results are shown in Figure 8.

The health evaluation model for sports individuals proposed in this paper can accurately predict the exercise limits of sports individuals and provide reasonable exercise recommendations, as shown in the figure. Because the server database must store a large amount of medical care and rehabilitation knowledge, the system must be able to access data quickly. The user prescriptions generated by the platform will be automatically saved, and users will be able to rate these sports programs. Instead of constantly filling in follow-up data, the Web platform will display the excellent exercise prescription on the front page, allowing matching users to learn directly from it. Because the relational database is flawed, it is impossible to truly match well. Personalized sports scheme design also necessitates the active participation of users. In this case, the platform also designed the service of expert consultation, wherein athletes can send their own sports health data directly to experts, and more customers can refer to the sports prescriptions of successful cases.

The sports health management platform takes personal sports health data information recording as the fundamental starting point, realizes dynamic evaluation on the basis of personal sports health data analysis, and then provides personal sports health improvement schemes and plans, which is of great significance for improving people's sports health level.

The article "Construction of Sports and Health Data Resources and Transformation of Teachers' Orientation Based on Web Database" was retracted in 2023. Reasons: suspected computer-generated content; unreliable results or conclusions; concerns about the data; concerns about the results or conclusions.

## 5. Conclusions

The construction of sports resources is based on the individual's sports and living habits and the actual health status, with sports consultation and personal fitness assessment as the main means, fully understanding the individual's sports goals and needs, and providing personalized sports programs on this basis, so as to guide the individual's health behavior, and finally improve the individual's physical fitness and sports health. The sports and health data resource system based on the Web database is based on summarizing and accumulating existing systems, and it is an all-round and systematic comprehensive health management system that combines many factors related to students' health, such as health education, sports activities, family, and society. It classifies the main factors affecting students' health into three major aspects: society, school, and family. In this paper, through the construction of sports health data system, the function of sports intervention in physical education in the health management system is used to promote and improve students' health level. This system can delete or add dynamic changes; the prescription database is continuously expanded and gradually improved; exercise mode, exercise belt, exercise amount, exercise intensity, exercise frequency, and other details are displayed, if requested; and the selected items are displayed visually by the built-in mathematical statistics formula in the system. It can provide convenient information collection, physical fitness evaluation, quick personalized nutrition prescription and exercise prescription output, and instant dietary nutrition evaluation, leading to an effective and convenient management platform for students' physical health promotion.

## Figures and Tables

**Figure 1:** Access process of web server.

**Figure 2:** System function module structure diagram.

**Figure 3:** Comparison of health status between students who participated in health management and those who did not.

**Figure 4:** Convergence curve of the algorithm.

**Figure 5:** Multi-thread server performance test results.

**Figure 6:** System server concurrent performance test results.

**Figure 7:** Comparison between energy consumption rate and limit energy consumption rate.

**Figure 8:** Error diagram of suggested time and actual time of the health evaluation model.

The article "Construction of Sports and Health Data Resources and Transformation of Teachers' Orientation Based on Web Database" was retracted in 2023. Reasons: suspected computer-generated content; unreliable results or conclusions; concerns about the data; concerns about the results or conclusions.

## Data Availability

The data used to support the findings of this study are included within the article.
